RETRACTED

# Pramipexole Inhibits Neuronal Apoptosis in Rats with Parkinson's Disease

**DOI:** 10.1155/2022/7002630

**Published:** 2022-04-13

**Authors:** Yongqi Sun, Baohong Cui, Lin Ye, Yunxin Hu, Yujun Pan

**Affiliations:** ^1^Department of Neurology, Guangdong 999 Brain Hospital, Guangzhou, China; ^2^Laboratory Medicine, The Third Affiliated Hospital of Harbin Medical University, Harbin, China; ^3^Department of Rehabilitation, Xuanwu Hospital Affiliated to Capital Medical University, Beijing, China; ^4^Department of Neurology, The First Affiliated Hospital of Harbin Medical University, Harbin, China

## Abstract

To explore the inhibition of pramipexole on the neuronal apoptosis and its influences on the expressions of brain tissue brain-derived neurotrophic factor (BDNF), and serum miR-103a and miR-30b and inflammatory factors in rats with Parkinson's disease. A total of 36 Sprague-Dawley rats were randomly divided into normal group (*n* = 12), model group (*n* = 12) and pramipexole group (*n* = 12). Compared with that in normal group, the positive expression of BDNF was substantially increased in model group and pramipexole group, and its positive expression in pramipexole group was notably higher than that in model group. The WB results revealed that compared with those in normal group, the relative protein expression levels of Bax and Bcl-2 were markedly increased and decreased, respectively, in the other two groups, and that pramipexole group exhibited a remarkable decline in the relative protein expression level of Bax and a considerable increase in that of Bcl-2, compared with model group. The relative expression levels of miR-103a and miR-30b in model and pramipexole groups were markedly higher than those in normal group, and pramipexole group had remarkably higher relative expression levels of miR-103a and miR-30b than model group. It was found through ELISA that model and pramipexole groups had markedly raised IL-1*β* and IL-18 content compared with normal group, and their content in pramipexole group was remarkably lower than that in model group. Based on the TUNEL results, compared with that in normal group, the apoptosis rate of cells rose substantially in the other two groups, and the apoptosis rate in pramipexole group was notably lower than that in model group. Pramipexole may up-regulate the expressions of BDNF, miR-103a and miR-30b to inhibit the apoptosis and inflammation in Parkinson's disease model rats.

## 1. Introduction

Parkinson's disease, one of clinically common central nervous system degenerative diseases and current difficulties in neurological treatment, is the most common in the middle-aged and elderly, and can cause such symptoms as muscle rigidity, tremor and autonomous motor dysfunction to patients, and as the disease progresses, the patients will further experience a series of extrapyramidal damage symptoms, including physical imbalance and muscle rigidity [1, 2].

RETRACTED

The current studies have demonstrated that [3–5] the major pathological mechanism is that the dopaminergic neurons are damaged, resulting in degeneration and loss, and further causing language and limb motor dysfunctions in the central nervous system. Thus, neuronal apoptosis and inflammation, as the leading pathological reactions, have been considered to have vital effects on Parkinson's disease. Additionally, brain-derived neurotrophic factor (BDNF), an important neurological factor in organisms, has been discovered to play a vital role in the repair of neurons and nervous system after Parkinson's disease [6], and the non-coding ribonucleic acids (RNAs) micro RNA (miR)-103a and miR-30b regulate several downstream signaling pathways to have important effects on neuronal apoptosis, inflammation and cell proliferation as well. As such, regulating these pathways may produce favorable efficacy in Parkinson's disease.

The purpose of the present study was to explore the effects of pramipexole on Parkinson's disease in rat models and to further investigate the potential mechanism.

## 2. Materials and Methods

### 2.1. Laboratory Animals and Grouping

A total of 36 Sprague-Dawley rats weighing (200 ± 20) g [Shanghai SLAC Laboratory Animal Co., Ltd., license No.: SCXK (Shanghai, China) 2014-0003] were assigned into normal group (*n* = 12), model group (*n* = 12) and pramipexole group (*n* = 12) using a random number table. The rat Parkinson's disease model was prepared through injecting rotenone-containing sunflower oil as follows: The rotenone-containing sunflower oil was subcutaneously injected into the neck of rats at a daily dose of 0.01 mL/kg, and the model could be established after continuous injection for 2 weeks [7].

### 2.2. Treatment in Each Group

The rats in normal group were normally fed, without any treatment, and after the Parkinson's disease model was prepared as above, those in model group and pramipexole group were intraperitoneally injected with an equal amount of normal saline and 0.05 mg/kg pramipexole daily, respectively. Following intervention for 7 d, the materials were sampled from each group.

### 2.3. Sampling

Upon successful anesthesia, abdominal aortic blood was drawn from all the rats. Then 6 rats in each group were perfused and fixed with paraformaldehyde, and brain tissues were obtained, fixed in 4% paraformaldehyde at 4°C for 48 h, and prepared into paraffin-embedded tissue sections for immunohistochemistry detection. Besides, the brain tissues of the remaining 6 rats in each group were directly taken and placed in EP tubes for Western blotting (WB) and qPCR.

RETRACTED

### 2.4. Immunohistochemistry

The tissues embedded in paraffin earlier were made into 5 *μ*m-thick sections, placed in 42°C warm water for extending, mounted, baked and prepared into paraffin-embedded tissue sections. Then they were routinely de-paraffinized and dehydrated through soaking in xylene solution and gradient ethanol successively. Subsequently, the resulting sections were immersed in citrate buffer and heated repeatedly using a micro-wave oven for 3 times (heating for 3 min and braising for 5 min per time) for complete antigen retrieval. After rinsing, the tissue sections were added dropwise with endogenous peroxidase blocker, reacted for 10 min, rinsed and sealed in goat serum for 20 min. With the goat serum sealing solution discarded, the tissue sections were incubated with the anti-BDNF primary antibody (1 : 200) in a refrigerator at 4°C overnight. On the next day, the rinsed sections were added dropwise with the secondary antibody solution, reacted for 10 min, fully rinsed, reacted with streptomycin avidin-peroxidase solution in drops for 10 min and added dropwise with DAB for color development. Finally, cell nuclei were counterstained using hematoxylin, and the sections were sealed and observed.

### 2.5. WB

The cryopreserved brain tissues were added with lysis buffer, bathed on ice for 1 h and then centrifuged at 14,000 g in a centrifuge for 10 min, followed by protein quantification using bicinchoninic acid (BCA) (Pierce, Rockford, IL, USA). The absorbance of proteins was measured using a microplate reader and the standard curve was plotted so as to calculate the concentration of proteins in the tissues. Subsequently, the proteins were denaturalized and isolated *via* sodium dodecyl sulphate-polyacrylamide gel electrophoresis (SDS-PAGE), until the marker protein was observed to be at the bottom of the glass plate like a straight line. The resulting proteins were transferred onto a polyvinylidene fluoride (PVDF) membranes (Roche, Basel, Switzerland), added with the sealing solution, reacted for 1.5 h and incubated successively with the anti-Bax primary antibody (1 : 1,000), anti-Bcl-2 primary antibody (1 : 1,000) and secondary antibodies (1 : 1,000). Finally, the proteins were reacted with chemiluminescent reagent for 1 min in the dark for complete image development.

### 2.6. QPCR

Total RNAs were first extracted and reversely transcribed into complementary DNAs (cDNAs) using the reverse transcription kit. Then qPCR was conducted in a reaction system (20 *μ*L) as follows: reaction at 51°C for 2 min, pre-degeneration at 96°C for 10 min, degeneration at 96°C for 10 s, and annealing at 60°C for 30 s, for 40 cycles. The relative expression levels of the related messenger RNAs (mRNAs) were calculated with glyceraldehyde-3-phosphate dehydrogenase (GAPDH) as an internal reference. The primer sequences are shown in Table 1.

RETRACTED

### 2.7. ELISA

The abdominal aortic blood was centrifuged at 14,000 g in a high-speed centrifuge for 10 min, and the supernatant was obtained. Then according to the instructions of the ELISA kit, the samples and standard were separately loaded into a plate and added with biotinylated antibody working solution and enzyme-conjugated substance working solution, and the plate was washed. Finally, the products were detected at 450 nm in the microplate reader.

### 2.8. TUNEL Apoptosis Assay

TUNEL assay was performed according to a previous report [8]. The pre-paraffin-embedded tissues were sliced into 5 *μ*m-thick sections, extended in warm water at 42°C, mounted, baked and prepared into paraffin-embedded tissue sections. Then these sections were routinely de-paraffinized and hydrated through immersing in xylene solution and gradient ethanol successively. Subsequently, the resulting sections were added dropwise with TdT reaction solution for reaction in the dark for 1 h, and incubated with deionized water in drops for 15 min to terminate the reaction. After the activity of endogenous peroxidase was blocked by adding hydrogen peroxide in drops, the sections were added dropwise with working solution. Following reaction for 1 h, the resulting sections were rinsed, added with diaminobenzidine (DAB) solution (Solarbio, Beijing, China) in drops for color development, rinsed again, sealed and observed.

### 2.9. Statistical Analysis

In this study, Statistical Product and Service Solutions (SPSS) 20.0 software (IBM, Armonk, NY, USA) was employed for statistical analysis, and enumeration data were expressed as mean ± standard deviation. *t*-test was performed for data conforming to normal distribution and homogeneity of variance, corrected *t*-test for those meeting normal distribution and heterogeneity of variance, and nonparametric test for those not in line with normal distribution and homogeneity of variance. Ranked data and enumeration data were subjected to rank sum test and chi-square test, respectively.

## 3. Results

### 3.1. Immunohistochemistry Results

Compared with that in normal group, the average optical density of cells with positive expression of BDNF rose substantially in model and pramipexole groups, showing a statistically significant difference (*P* < 0.05), and the average optical density in pramipexole group was higher than that in model group, with a statistically significant difference (*P* < 0.05) (Figure 1).

RETRACTED

### 3.2. Pramipexole Reduced Bax and Increased Bcl-2

Normal group had fewer expressed Bax proteins and more expressed Bcl-2 proteins than the other two groups (Figure 2). The statistical results revealed that compared with those in normal group, the relative protein expression levels of Bax and Bcl-2 were markedly increased and decreased, respectively, in the other two groups (*P* < 0.05), and that pramipexole group showed a remarkably lower relative protein expression level of Bax and a considerably higher relative protein expression level of Bcl-2 than model group (*P* < 0.05).

### 3.3. Higher Levels of miR-103a and miR-30b after Pramipexole Treatment

As shown in Figure 3, compared with normal group, model and pramipexole groups exhibited substantial increases in the relative expression levels of miR-103a and miR-30b, with statistically significant differences (*P* < 0.05). Besides, the relative expression levels of miR-103a and miR-30b in pramipexole group were notably higher than those in model group, and the differences were statistically significant (*P* < 0.05).

### 3.4. Pramipexole Reduced IL-1*β* and IL-18

Compared with that in normal group, the content of IL-1*β* and IL-18 was remarkably elevated in model and pramipexole groups, showing a statistically significant difference (*P* < 0.05), and their content in pramipexole group declined remarkably in comparison with that in model group, displaying a statistically significant difference (*P* < 0.05) (Figure 4).

### 3.5. Pramipexole Inhibited Apoptosis

Apoptotic cells were tan, and normal group had fewer apoptotic cells than the other two groups. Compared with normal group, the other two groups exhibited a substantial increase in the average optical density of TUNEL-positive apoptotic cells, showing a statistically significant difference (*P* < 0.05), and the average optical density in pramipexole group was notably higher than that in model group, with a statistically significant difference (*P* < 0.05) (Figure 5).

## 4. Discussion

Parkinson's disease is one of the most common degenerative diseases in the central nervous system in clinic, and as a nervous system disease frequently occurring in the elderly, it has high morbidity and disability rates, seriously affecting the living quality and life health, so there is an urgent need for its further research. As the research of Parkinson's disease progresses, it has been recognized by researchers that the most important pathological reaction mechanism of Parkinson's disease is extrapyramidal injury that further causes a series of cascade reactions, such as inflammation, neuronal apoptosis and necrosis [9]. Hence, the relevant pathogenesis of Parkinson's disease remains very complex and elusive. Studies have demonstrated that [10, 11] after the extrapyramidal system is damaged, the pathological reactions in extrapyramidal neurons, such as apoptosis, necrosis and inflammation will be induced by multiple factors, including cytokines, inflammatory factors, and oxidative stress responses to further aggravate extrapyramidal injury, and ultimately result in the degeneration and loss of neurons in the central nervous system, which is not conducive to the post-injury repair. Additionally, BDNF, as one member in the vital neurotrophic factor family, has important effects on the repair and regeneration of the nervous system, such as neuronal regeneration, axon regeneration, and synaptic myelination, which is a crucial substance in the field of the central nervous system diseases [12–15]. Therefore, the related treatment of Parkinson's disease is still one of the hotspots and difficulties in the clinical and basic research fields. According to several studies [16, 17], raising the content of BDNF in the local damaged central nervous system can effectively promote the regeneration of neurons and axons in the local central nervous system, reconstruction of nervous system networks and reconnection of synapses and dendrites, thereby producing vital effects and influences on the repair of the central nervous system. Therefore, BDNF has become a target for the repair of the central nervous system, and effective enhancement of its expression after injury significantly accelerates the repair of the nervous system, further improving the behavioral characteristics of the Parkinson's disease model rats. As non-coding RNAs, both miR-103a and miR-30b play important roles in neuronal apoptosis, inflammation and cell proliferation through regulating several downstream signaling pathways as well. They modulate the downstream target gene transcription and target protein translation to resist inflammation and apoptosis, thus benefiting the post-injury repair [18–20], so miR-103a and miR-30b have gradually been regarded as the important action targets for the treatment of the central nervous system diseases.

RETRACTED

According to the results of this study, the brain tissues of the Parkinson's disease model rats had excessive neuronal inflammation and apoptosis, which may be one cause of Parkinson's disease. Moreover, after the onset of Parkinson's disease, the aberrantly high expressions of BDNF, miR-103a and miR-30b were detected, indicating that all of them serve as important players in the onset of Parkinson's disease. Pramipexole, a clinically common drug for treating Parkinson's disease, has favorable inhibitory effects on the neuronal inflammation and apoptosis in the brain tissues of the Parkinson's disease model rats, while effectively up-regulating the expressions of BDNF, miR-103a and miR-30b, which is likely to be one mechanism of pramipexole in treating Parkinson's disease. Therefore, it can be known that pramipexole may up-regulate the expressions of BDNF, miR-103a and miR-30b to inhibit the apoptosis and inflammation in the Parkinson's disease model rats.

Limitations existed in the current study. We found that the relative expression levels of miR-103a and miR-30b in pramipexole group were notably higher than those in model group, however, we did not perform the further experiments to explore why pramipexole can increase the levels of miR-103a and miR-30b. Additionally, the role of miR-103a and miR-30b in Parkinson's disease should also be further investigated by future studies.

## 5. Conclusions

Therefore, it can be known that pramipexole may up-regulate the expressions of BDNF, miR-103a and miR-30b to inhibit the apoptosis and inflammation in the Parkinson's disease model rats.

## Figures and Tables

**Figure 1:** BDNF expression detected *via* immunohistochemistry. Comparison of positive expression of BDNF among all groups. Note: ^*∗*^*P* < 0.05*vs.* normal group, and ^#^*P* < 0.05*vs.* model group.

**Figure 2:** Relative expression levels of bax and Bcl-2 in each group. Note: ^*∗*^*P* < 0.05 vs. normal group, and ^#^*P* < 0.05*vs.* model group.

**Figure 3:** Expressions of miR-103a and miR-30b among all groups. Note: ^*∗*^*P* < 0.05 vs. normal group, and ^#^*P* < 0.05*vs*. model group.

**Figure 4:** Levels of inflammatory factors (IL-1*β* and IL-18) in each group. Note: ^*∗*^*P* < 0.05 vs. normal group, and ^#^*P* < 0.05*vs.* model group.

**Figure 5:** Cell apoptosis detected *via* TUNEL assay. Comparison of cell apoptosis rate among all groups. Note: ^*∗*^*P* < 0.05*vs*. normal group, and ^#^*P* < 0.05 vs. model group.

**Table 1:** List of primer sequences.

Name	Primer sequence
MiR-103a	Forward: 5′ TCTTTCCAGATGAACAAATGGC 3′ Reverse: 5′ GCTGTTTTTCGCTTGAAATCTGC 3′

MiR-30b	Forward: 5′TTCCTAGTGTTGACGAATCTTGC 3′ Reverse: 5′GCAGACAGGACCTGTAATCTGG 3′

GAPDH	Forward: 5′ ACGGCAAGTTCAACGGCACAG 3′ Reverse: 5′ GAAGACGCCAGTAGACTCCACGAC 3′

## Data Availability

The datasets used and analyzed during the current study are available from the corresponding author on reasonable request.
